The article "A Novel Three-Dimensional Immune Oncology Model for High-Throughput Testing of Tumoricidal Activity" was published in 2018. Journal: Front Immunol.

# A Novel Three-Dimensional Immune Oncology Model for High-Throughput Testing of Tumoricidal Activity

**DOI:** 10.3389/fimmu.2018.00857

**Published:** 2018-04-23

**Authors:** Hilary Sherman, Hannah J. Gitschier, Ann E. Rossi

**Affiliations:** Life Sciences Division, Corning Incorporated, Kennebunk, ME, United States

**Keywords:** cancer, immune cell invasion, immune cell infiltration, immune cell migration, immune oncology, spheroid, three-dimensional cell culture, transwell

## Abstract

The latest advancements in oncology research are focused on autologous immune cell therapy. However, the effectiveness of this type of immunotherapy for cancer remediation is not equivalent for all patients or cancer types. This suggests the need for better preclinical screening models that more closely recapitulate *in vivo* tumor biology. The established method for investigating tumoricidal activity of immunotherapies has been study of two-dimensional (2D) monolayer cultures of immortalized cancer cell lines or primary tumor cells in standard tissue culture vessels. Indeed, a proven means to examine immune cell migration and invasion are 2D chemotaxis assays in permeabilized supports or Boyden chambers. Nevertheless, the more *in vivo*-like three-dimensional (3D) multicellular tumor spheroids are quickly becoming the favored model to examine immune cell invasion and tumor cell cytotoxicity. Accordingly, we have developed a 3D immune oncology model by combining 96-well permeable support systems and 96-well low-attachment microplates. The use of the permeable support system enables assessment of immune cell migration, which was tested in this study as chemotactic response of natural killer NK-92MI cells to human stromal-cell derived factor-1 (SDF-1α). Immune invasion was assessed by measuring NK-92MI infiltration into lung carcinoma A549 cell spheroids that were formed in low-attachment microplates. The novel pairing of the permeable support system with low-attachment microplates permitted simultaneous investigation of immune cell homing, immune invasion of tumor spheroids, and spheroid cytotoxicity. In effect, the system represents a more comprehensive and *in vivo*-like immune oncology model that can be utilized for high-throughput study of tumoricidal activity.

## Introduction

Harnessing the power of the immune system *via* immunomodulatory and/or cell-based therapeutics holds great promise and is a very active area of both academic and clinical oncology research. In the simplest terms, cancer immunotherapies take advantage of patients’ own immune responses either by boosting the natural response to tumor antigens or by directing specific attack on malignant cells (1–3). Yet, some promising cancer immunotherapies have fallen short in a clinical setting (1). This highlights the need for improved *in vitro* screening methods that yield results more predictive of clinical efficacy.

The article "A Novel Three-Dimensional Immune Oncology Model for High-Throughput Testing of Tumoricidal Activity" was published in 2018. Journal: Front Immunol.

Traditionally, tumoricidal activity and immune evasion have been studied by utilizing two-dimensional systems (2D). In 2D systems, either immortalized cancer cell lines or primary tumor cells are cultured as a monolayer on standard tissue culture vessels. Primary testing *via* 2D methods is often the entry point into preclinical drug screening cascades. Yet, these 2D models do not accurately reflect the complexity of a three-dimensional (3D) tumor (4), a characteristic that has been cited as a contributing factor to the high attrition rate of cancer drugs (5, 6). The most obvious difference between 2D culture and a 3D system is the architecture of the collection of cells. The context provided by a 3D environment affects the nature of cell–cell contacts and the formation of extracellular matrix surrounding the cells. Structural complexity of spheroids creates more physiological barriers to immune cells (versus 2D culture). As *in vivo*, the immune cells need to infiltrate the 3D cell-matrix formation in order to attack the malignant target cells (4, 7–9). Furthermore, tumor cells cultured in 3D more closely mimic *in vivo* tumor biology in terms of signaling (4, 8, 9). For example, it has been shown that phenotypic differences occur in 3D-cultured tumor cells that allow for higher resistance to cytotoxicity. In a 2003 study, Dangles-Marie et al. found a decrease in Hsp70 and subsequent decrease in antigen presentation in 3D culture of a lung carcinoma cell line (IGR-Heu). Diminished antigen presentation rendered the cells less susceptible to cytotoxic T lymphocyte attack (10). Similarly, there is a threshold effect of MHC Class-I expression in 3D spheroids of Ewing’s sarcoma tumor (ESFT) cells. This tips the balance of natural killer (NK) cell signaling toward inhibitory inputs, allowing NK evasion by ESFT spheroids (11). Many other examples of the morphological (12) and phenotypic (13–15) differences between 2D and 3D experimental cell culture models have been published in the primary literature making it clear that 3D tumor models more closely resemble the *in vivo* tumor microenvironment.

Thus, 3D cell culture provides more physiological disease modeling. Improving *in vitro* oncology models by utilizing 3D cell culture will create screening tools with greater accuracy in assessing therapeutic efficacy. To this end, we demonstrate a high-throughput 3D model to study cancer/immune cell interactions by a novel combination of two commercially available products: 96-well permeable support systems and 96-well ultra-low-attachment microplates. By replacing the standard 2D flat-bottom permeable support receiver plate with an ultra-low-attachment microplate, we have created an easy-to-use, 3D high-throughput assay to investigate immune cell homing, tumor cytotoxicity, and tumor immune evasion.

The article "A Novel Three-Dimensional Immune Oncology Model for High-Throughput Testing of Tumoricidal Activity" was published in 2018. Journal: Front Immunol.

## Materials and Methods

### Immune Cell Migration

NK-92MI (ATCC^®^ Cat. No. CRL-2408) cells were cultured in Iscove’s Modification of DMEM (IMDM; Corning Cat. No. 10-016-CM) supplemented with 10% fetal bovine serum (FBS, Corning Cat. No. 35-010-CV). Before seeding for the migration assay, cells were stained by incubation with 80 µM CellTracker™ Blue CMHC Dye (Molecular Probes™ Cat. No. C2111) in IMDM for 1 h. After labeling, 1.5 × 10^5^ cells in 100 µL were added to each insert of a Corning^®^ HTS Transwell^®^-96 Tissue Culture System (Corning Cat. No. 3387) and allowed to migrate overnight (16–24 h) toward various concentrations of human stromal-cell derived factor-1 (SDF-1α)/CXCL12 (Shenandoah Biotechnology Inc.™ Cat. No. 100-20) in IMDB + 10% FBS. Vehicle control (IMDM + 10% FBS) was included to determine passive migration. We anticipated there would be only 5% or less migration at low doses of SDF-1α and chose to use a high cell density to ensure there would be a sufficient number of cells to enumerate. Migration was quantified by measuring Cell Tracker™ Blue fluorescence *via* flow cytometry using the Miltenyi Biotec MacsQuant^®^ and expressed as a ratio of cells in basolateral chamber compared with total cells seeded in insert.

### Tumor Spheroid Formation and Immune Infiltration

Lung carcinoma A549/GFP cells (Cell Biolabs, Inc. Cat. No. AKR-209), were seeded into 96-well spheroid microplates (Corning Cat. No. 4515) at 2 × 10^3^ cells/well in 100 µL of IMDM + 10% FBS. The plate was incubated 24 h at 37°C, 5% CO_2_ which was sufficient to form spheroid structures. After spheroid formation, 100 µL of varying concentrations of effector cells (5 × 10^2^–3.2 × 10^4^ cells) were added to A549 spheroids for overnight incubation. We used both NK-92MI and MOLT-4 (ATCC Cat. No. CRL-1582) cells pre-labeled with CellTracker™ Blue CMHC Dye. Morphology of the spheroid with NK-92MI infiltration was examined by immunohistochemical staining of the leukocyte marker CD45 (Abcam Cat. No. ab40763) and endothelial marker e-cadherin (Abcam Cat. No. ab1416). Spheroids were fixed in 4% paraformaldehyde and paraffin embedded before sectioning and staining for 1 h in anti-CD45 at 1:100 (6.3 µg/mL) and anti-e-cadherin at 1:200 (1.9 µg/mL). Detection was performed using the Enzo Multiview HRP/AP kit (Enzo Life Sciences Cat. No. ADI-950-100-0001) according to manufacturer’s instructions. Nuclei were counterstained with hematoxylin. The impact of effector cell type and number on the spheroids was assessed by analyzing the dissociated spheroid. Briefly, culture medium was removed and replaced with 150 µL 10X TrypLE™ Select Enzyme (10×) (Gibco™ Cat. No. A1217701). Spheroids were incubated at 37°C until they could be broken up into single cells with minimal pipetting (~20 min). Fluorescence of the dissociated cells was quantified *via* flow cytometry, gating for GFP and CellTracker Blue fluorescence. Gating was set to high GFP fluorescence, minimizing the contribution of GFP-positive apoptotic cells, so that GFP-positive cell count was used as a surrogate for cell viability. A549 percent cytotoxicity was calculated relative to A549 cell count in the absence of effector cells.

The article "A Novel Three-Dimensional Immune Oncology Model for High-Throughput Testing of Tumoricidal Activity" was published in 2018. Journal: Front Immunol.

### 3D Immune Oncology Model

A549/GFP cells (2 × 10^3^ cells/well) were seeded into 96-well spheroid microplates. The next day, medium was replaced with 200 µL of IMDM + 10% FBS containing 3.75 nM of SDF or vehicle control (IMDM+10% FBS). NK92-MI cells were stained as previously described while simultaneously being treated with 5.7 µM prostaglandin E2 (PGE_2_; Tocris Cat. No. 2296) dissolved in IMDM or vehicle control (IMDM) for 1 h. HTS Transwell-96-Well Permeable Supports were placed in 96-well spheroid plates (a schematic is shown in Figure 1). NK-92MI cells were then resuspended in serum-free IMDM and seeded into inserts at 5 × 10^4^ cells/well. To account for non-migratory cells, NK-92MI cells were seeded in excess of the number required for direct cytotoxicity assay. After 24 h, inserts were removed, and spheroid microplates were processed for flow cytometry to calculate percent migration of NK92-MI cells and A549 percent viability.

**Figure 1:** Assay diagram. GFP-labeled A549 cells are cultured in 96-well ultra-low-attachment microplates to generate tumor spheroids. The spheroid microplate then becomes the receiver for 96-well Transwell inserts, into which CellTracker™ Blue-labeled NK-92MI are seeded. The plates are incubated together to allow for natural killer cell migration, invasion of the spheroid and subsequent cytotoxicity.

### Statistics

All data graphed as mean ± SD. Statistical significance determined by one- or two-way ANOVA with Bonferroni *post hoc* test using GraphPad Prism.

## Results and Discussion

### Migration

An important component to any immune response is the activation of immune cells and subsequent relocation to the target area requiring defense. *In vitro* migration studies allow for evaluating immune cell recruitment to determine conditions which enhance or suppress this activity. In this study, cells from a NK cell line derived from peripheral blood, NK-92MI, were placed in the apical compartments of Transwell inserts with 5.0-µm pore size, and allowed to migrate overnight toward medium containing various concentrations of SDF-1α, a CXC chemokine that signals through the CXCR4 receptor and known chemoattractant for lymphocytes (16). In the absence of SDF-1α, there was a 2.5% average passive migration (Figure 2). The concentration response curve for NK-92MI chemotaxis generated an EC_50_ value of 1.76 nM, which is consistent with values for NK cell lines and primary NK cell chemotaxis reported in literature (17).

The article "A Novel Three-Dimensional Immune Oncology Model for High-Throughput Testing of Tumoricidal Activity" was published in 2018. Journal: Front Immunol.

**Figure 2:** Dose-dependent migration of NK-92MI cells toward stromal-cell derived factor-1 (SDF-1α). NK-92MI (NK) cells were evaluated for migration to varying concentrations of chemokine SDF-1α. Cells in basolateral chambers were quantified by flow cytometry. Data are plotted as the ratio of migration induced by chemokine compared with total cells seeded in insert. Average% migration in the absence of SDF-1α is plotted as a dotted line with the mean ± SD range indicated as ticks on the left axis, *n* = 6 wells. Data represent the average of two independent studies, *n* = 24 wells.

### Infiltration

The presence of certain immune cells in a malignant structure has been shown to correlate with increased patient survival (18). To this end, 3D models can be utilized to observe immune cell infiltration into the spheroid unlike more commonly used 2D *in vitro* models for studying immune cytotoxicity. Two common methodologies for visualizing immune cell infiltration are histology and confocal microscopy. Figure 3A shows e-cadherin (brown) and CD45 (red) stained sections of A549/GFP spheroids infiltrated by NK-92MI cells. Infiltration can also be observed *via* confocal microscopy as shown in Figure 3B, with noticeable blue NK-92MI cells interspersed with the green A549/GFP cells of the spheroid. The appearance of a larger spheroid is consistent with breakup of the spheroid architecture resulting from the cytotoxic effect of infiltrating NK cells. These studies confirm that the immune cells in this model are not only able to reach the target tumor cells, but are also capable of infiltrating the 3D spheroid structure.

**Figure 3:** NK-92MI cell infiltration into A549/GFP tumor spheroids. **(A)** Representative histological sections of CD45- (red) and e-cadherin-stained (brown) of A549/GFP spheroids (*left*) and spheroids exposed to NK-92MI cells for 4 h (*right*) at 200× magnification. **(B)** Maximum projection confocal images of A549/GFP spheroids (green) subjected to NK-92MI cell (blue) infiltration. Images taken at 20× with a Z stack height of 125 µm *via* Thermo Scientific™ CellInsight™ CX7. Scale bars are 100 µm **(A)** and 200 µm **(B)**.

The article "A Novel Three-Dimensional Immune Oncology Model for High-Throughput Testing of Tumoricidal Activity" was published in 2018. Journal: Front Immunol.

### 3D Cytotoxicity

To investigate the immune-induced cytotoxicity of A549 cells, both NK-92MI and MOLT-4 suspension cells were added to spheroid microplates containing preformed A549 tumor spheroids. NK92-MI cells are known to be cytotoxic to a wide range of malignant cells. MOLT-4 cells were used as a negative control because they are a T-cell leukemia cell line with no known cytotoxic effect on other malignant cells. Figure 4 demonstrates the dose-dependent effect NK-92MI cells on A549/GFP viability, in contrast to the limited effect of MOLT-4 cells which only show toxicity show at the highest concentrations. These data support the specific targeting of the NK-92MI cells to the A549 cells and resulting tumor spheroid cell death.

**Figure 4:** Specific and dose-dependent effector function demonstrated by NK-92MI cells. NK-92MI (NK, green) cells added at various concentrations to A549/GFP (A549) tumor spheroids displayed dose-dependent cytotoxicity that was significantly left-shifted compared with that observed with MOLT-4 cells (black), a T-cell leukemia cell line with no known cytotoxic effect on other malignant cells (*p* < 0.0051, two-way ANOVA). Data represent the average of two independent studies, *n* = 12 wells per concentration.

### Migration With Cytotoxicity

To evaluate the migration and cytotoxic effects of immune cells on tumor spheroids in 3D in one single, easy-to-use high-throughput assay, the HTS Transwell^®^-96 Tissue Culture System and spheroid microplate were combined as previously described (Figure 1). As MOLT-4 cells did not induce appreciable cytotoxicity, the paired migration/infiltration model was examined with NK-92MI cells. Figure 5 demonstrates how NK cell migration can be enhanced by the addition of chemokines, such as SDF-1α, as well as suppressed by the addition of inhibitors, such as PGE_2_. NK migration was significantly increased when the chemoattractant SDF-1α was present in the receiver or spheroid microplate. Conversely, migration was significantly decreased when NK cells were exposed to PGE_2_, a known inhibitor of immune cell function that is often secreted by cancer cells as a form of immune evasion (19). Notably, tumoricidal activity corresponds well with migration data, with high migration associated with high levels of cytotoxicity. Specifically, the highest % cytotoxicity and highest % migration values were observed with NK cells exposed to SDF. Addition of PGE_2_ to inhibit NK cell migration resulted in decreased A549 cytotoxicity relative to SDF alone (Figure 5).

The article "A Novel Three-Dimensional Immune Oncology Model for High-Throughput Testing of Tumoricidal Activity" was published in 2018. Journal: Front Immunol.

**Figure 5:** NK-92MI cell migration and subsequent cytotoxicity toward A549/GFP spheroids. NK-92MI (NK) cell migration (blue) was evaluated in the presence and absence of stromal-cell derived factor-1 (SDF-1α) and/or prostaglandin E2 (PGE) in the medium. Percent migration (left axis) was calculated as a ratio of cells in basolateral chamber compared with total cells seeded in insert. Cytotoxicity of A549/GFP cells (green) was evaluated after exposure to NK-92MI (NK) cells in the presence and absence of SDF-1α and/or PGE in the medium. Percent viability (right axis) was calculated *via* flow cytometry by enumerating GFP-positive A549 cells relative to spheroids without effector cells. Data are shown as the average of two independent studies, *n* = 24 wells. *p < 0.001 and **p < 0.0001 in one-way ANOVA with Bonferroni *post hoc* test.

## Conclusion

In order to create a model system to investigate immune cell homing, 3D tumor cytotoxicity, and tumor immune invasion in a single, high-throughput assay, we combined a 96-well low-attachment microplate and a 96-well permeable support system. Previous studies have investigated separate components of this model by looking at either cell migration from a 2D cell monolayer (20–22) or 3D tumoricidal activity independent of immune cell homing (8, 10, 11, 20, 23). Commonly, Transwell-based assays (permeable supports or Boyden chambers) are employed to study migration of cells in 2D in response to chemotactic gradients (20–22). Invasion assays are an extension of the Transwell assay in which a thin layer of matrix occludes the pores of the permeable membrane to prevent non-invasive cells from migrating through the membrane. Transwell migration/invasion assays have well-established protocols and are excellent endpoint methods to study cell homing and invasion (7, 20, 24). Yet, they lack the complex physiology of 3D cell cultures.

Though sometimes more difficult to implement, studies utilizing spheroids more closely mimic the tumor microenvironment and can recapitulate tumoricidal activity seen *in vivo* (7–11, 25). For example, Herter et al. reconstituted the heterogenous cell populations of *in vivo* tumors by creating heterotypic spheroids of human colon adenocarcinoma cells, fibroblasts, and peripheral blood mononuclear cells (PBMCs) (9). Treatment of the spheroids with an interleukin-2 variant (IgG-IL2v) and carcinoembryonic antigen-targeted T-cell bispecific antibody (CEA-TCB) activated T, NK and NK T cells, and enhanced immune cell invasion into the spheroids (9). Similarly, Giannattasio et al. presented a human cervical carcinoma spheroid model susceptible to NK cell invasion and cytotoxicity (8). Tumor spheroids were found to express NK-activating receptor ligands, making them a target for NK-mediated destruction. Consequently, primary NK cells were able to infiltrate spheroids and lyse the tumor cells, destroying the spheroid structure. Giannattasio et al. went on to demonstrate that just as tumor cells are capable of immune escape mechanism *in vivo*, the tumor spheroids shed NK-activating receptor ligands with prolonged spheroid culture (8). Importantly, tumor spheroids provided an added level of structural complexity within which to investigate 3D tumor cytotoxicity and tumor immune evasion.

The article "A Novel Three-Dimensional Immune Oncology Model for High-Throughput Testing of Tumoricidal Activity" was published in 2018. Journal: Front Immunol.

By exploiting the advantages of both 2D and 3D assays, we have developed a more comprehensive assay tool and a more *in vivo*-like immune oncology model. Although we describe the method with commonly used NK-92MI cells and a GFP-expressing A549 tumor cell line, the focus was not, *per se*, on the specific cell types. Rather, the goal of this study was to provide a framework from which to optimize for specific cells of interest. For example, there is utility in adapting this assay for primary murine cells. *Ex vivo* murine tissue samples and *in vivo* preclinical rodent model data that can be more attainable than human samples would be a ready comparison to validate physiological relevance of the system.

The data presented in this manuscript provide proof of concept. Transwell migration/invasion assays are well characterized and there are standardized protocols available. In addition, a wide variety of cell lines have been used to generate spheroids in spheroid microplates and the basic protocol remains the same. The exact formation, size, and duration of multicellular spheroid culture in the spheroid microplate are cell line dependent. Optimization of cell-seeding conditions for the formation of multicellular tumor spheroids of a desired size within a specified culture period is very straightforward. As a result, the method described would be amenable to assay numerous different target and effector cell types. The versatility of the novel pairing of the permeable support system with low-attachment microplates makes it a powerful tool for simultaneous assay of immune cell migration, invasion, and subsequent tumoricidal activity.

## Author Contributions

HS and HG were involved in study design. HS performed all experiments and analyzed data. HS and HG reviewed and compiled data and prepared the manuscript. AR edited and formatted manuscript for publication. All authors have read and approved final manuscript.

## Conflict of Interest Statement

All authors are employees by Corning Incorporated.
